# miR-136 Modulates TGF-*β*1-Induced Proliferation Arrest by Targeting PPP2R2A in Keratinocytes

**DOI:** 10.1155/2015/453518

**Published:** 2015-01-14

**Authors:** Dianbao Zhang, Jing Wang, Zhe Wang, Tao Zhang, Ping Shi, Xiliang Wang, Feng Zhao, Xiaoyu Liu, Xuewen Lin, Xining Pang

**Affiliations:** ^1^Department of Stem Cells and Regenerative Medicine, Key Laboratory of Cell Biology, Ministry of Public Health and Key Laboratory of Medical Cell Biology, Ministry of Education, China Medical University, Shenyang 110001, China; ^2^Department of Anus & Intestine Surgery, The First Affiliated Hospital, China Medical University, Shenyang 110001, China; ^3^Department of Blood Transfusion, Shengjing Hospital, China Medical University, Shenyang 110004, China; ^4^Department of General Practice, The First Affiliated Hospital, China Medical University, Shenyang 110001, China

## Abstract

Keratinocytes proliferation is critical for the capacity to heal wounds and accumulating evidences have proved that dysregulation of microRNAs is involved in proliferation of keratinocytes. However, the molecular mechanisms remain to be completely elucidated. Here, we show that miR-136 was significantly decreased by TGF-*β*1 treatment in HaCaT cells and normal human epidermal keratinocytes (NHEK), and it was a Smad3-dependent manner. By cell proliferation assay and cell cycle analysis, we found that reintroduction of miR-136 by transfection, as well as PPP2R2A silencing, counteracted TGF-*β*-induced proliferation arrest in HaCaT cells. Further, PPP2R2A was verified as a direct target of miR-136 by dual-luciferase reporter assays and Western blotting. These data suggest that miR-136 may play an important role during TGF-*β*1-induced proliferation arrest by targeting PPP2R2A in keratinocytes, which might represent a potential target for improving skin wound healing.

## 1. Introduction

Keratinocytes proliferation is essential for the formation of skin appendages and reepithelialization after wounding [1], and epidermal homeostasis depends on a balance of keratinocytes between proliferation in the basal layer and differentiation/apoptosis in the superbasal layer [2–4]. So far, these functions have been shown to be stimulated by many growth factors, including transforming growth factor-*β*1 (TGF-*β*1) [5, 6]. Moreover, TGF-*β*1 secreted by fibroblasts and keratinocytes would cause proliferation arrest of keratinocytes through activating the signaling pathways by binding a receptor complex comprising two transmembrane serine/threonine kinases known as the type I and type II receptors [7]. Thus, exploring the regulation mechanisms of TGF-*β*1-induced keratinocytes proliferation arrest is necessary to understand skin development and wound repair and to design novel therapeutic strategies for skin wound healing.

MicroRNAs (miRNAs) represent a large family of conserved noncoding small RNAs (~21 nucleotides long), which have emerged as key regulators of gene expression at both the transcriptional and translational levels. Recently, increasing evidences suggest that miRNAs are responsible for regulating proliferation and self-renewal of keratinocytes [8]. Depletion of the miRNA processing enzyme Dicer in the epidermis results in hyperproliferation [9], and several miRNAs have been shown to modulate keratinocytes proliferation, such as miR-34 family [10], miR-125b [11], miR-200 family [12], miR-203 [13], and miR-210 [14]. Nonetheless, the crucial role of miR-136 in the TGF-*β*1-induced proliferation arrest is largely unknown.

PPP2R2A, also known as B55*α*, is a regulatory subunit of the protein phosphatase 2A (PP2A), which is one of the four major serine/threonine (Ser/Thr) phosphatases, and is implicated in the negative control of cell growth and division in mammalian cells [15, 16]. The crystal structure of PPP2R2A has provided insight on how the B subunit forms a pocket with the catalytic subunit that may confer substrate specificity [17]. PPP2R2A plays an important role in the modulation of the phosphorylation state of pocket proteins and mitotic CDK substrates throughout the cell cycle and in quiescent cells [18].

In the present study, we identified and characterized PPP2R2A as a functional downstream target of miR-136 and examined the roles of miR-136 and PPP2R2A in TGF-*β*1-induced proliferation arrest in keratinocytes.

## 2. Materials and Methods

### 2.1. Cell Isolation and Culture

Normal human epidermal keratinocytes (NHEK) were isolated from foreskins (18–26 years old, *n* = 3) using Dispase II (Roche, IN, USA) to remove the dermis from the epidermis followed by trypsinization and culture in EpiLife serum-free medium with 60 *μ*M calcium supplemented with HKGS (Gibco, NY, USA). Written informed consent was obtained from all patients and approval of the China Medical University Ethics Committee was obtained.

The immortalized human keratinocyte cell line HaCaT was kindly provided by Chundi He. Cos-7 cells were purchased from ATCC. HaCaT cells and Cos-7 cells were cultured in DMEM (Hyclone, MA, USA) supplemented with 10% fetal bovine serum. All the cells were maintained under standard conditions at 37°C and 5% CO_2_ in a humid atmosphere. For TGF-*β*1 treatment, NHEK or HaCaT cells were plated at 3,000 cells/cm^2^ and maintained for 24 h, after which they were serum-starved for another 24 h. Then, the cells were cultured in the absence or presence of TGF-*β*1 (R&D Systems, MN, USA) for 48 h and 72 h.

### 2.2. Quantitative Real-Time PCR (qRT-PCR)

Total RNA was extracted using TRIzol reagents (Invitrogen, CA, USA) according to the manufacturer's protocol. To analyze miR-136 expression, reverse transcription PCR was performed using specific stem-loop RT primers from a Hairpin-it miRNAs qPCR Quantitation Kit (GenePharma, Shanghai, China), and quantitative real-time PCR was performed using the same kit on Applied Biosystems 7500 system. U6 was used as an internal control. To quantify mRNA level of PPP2R2A and Smad3, reverse transcription PCR was applied using PrimeScript RT Reagent Kit with gDNA Eraser (Takara, Dalian, China) and quantitative real-time PCR was performed using SYBR Premix Ex Taq (Takara, Dalian, China). GAPDH was used as an internal control. Fold changes of both miRNA and mRNA were calculated using the 2^−ΔΔCt^ method. Each experiment was performed in triplicate. The primer sequences were as follows: 5′-AACCCACTTCCTGCTTAGTTGAG-3′ (forward) and 5′-GAACACCACAGTGATGAATCCAC-3′ (reverse) for human PPP2R2A; 5′-ACTACATCGGAGGGGAGGTC-3′ (forward) and 5′-TGCATCCTGGTGGGATCTTG-3′ (reverse) for human Smad3; 5′-GCACCGTCAAGGCTGAGAAC-3′ (forward) and 5′-TGGTGAAGACGCCAGTGGA-3′ (reverse) for human GAPDH.

### 2.3. miRNA and siRNA Transfection

Cells cultured in 6-well plates were transfected at 30–50% confluence using Lipofectamine RNAiMAX Transfection Reagent (Invitrogen, CA, USA) with Opti-MEM I (Gibco, NY, USA) according to the manufacturer's instructions. Briefly, 25 pmol of miR-136 mimics, PPP2R2A siRNA (Santa Cruz, CA, USA), Smad3 siRNA, or negative control (NC) was used with 7.5 *μ*L of the transfection reagent and the medium was replaced with fresh medium 24 h after transfection. Smad3 siRNA, miR-136 mimics, and NC were chemical synthesized by GenePharma (Shanghai, China) and the sequences were as follows: 5′-GAGCCTGGTCAAGAAACTCAATT-3′ for Smad3 siRNA, 5′-ACUCCAUUUGUUUUGAUGAUGGA-3′ for miR-136 mimics, and 5′-UUCUCCGAACGUGUCACGUTT-3′ for NC.

### 2.4. Cell Proliferation Assay

Cell proliferation was measured using Cell Counting Kit-8 (CCK-8, Dojindo, Kumamoto, Japan). 10 *μ*L CCK-8 was added to cells maintained in 96-well plates and the cells were subsequently incubated for 2 h at 37°C. The absorbance of each sample at 450 nm was measured with a reference wavelength of 630 nm. All experiments were performed in triplicate and repeated three times.

### 2.5. Cell Cycle Analysis

Cell Cycle and Apoptosis Analysis Kit (Beyotime, Nantong, China) was used for cell cycle analysis. Cells were fixed in 70% ethanol in PBS at −20°C for 12 h after washing three times with cold PBS; then the cells were washed again and stained with 0.5 mL of propidium iodide (PI) staining buffer (it contains 200 mg/mL RNase A and 50 *μ*g/mL PI) at 37°C for 30 min in the dark. Analyses were performed on BD LSR flow cytometer. The experiments were repeated three times.

### 2.6. Dual-Luciferase Reporter Assays

Bioinformatic analysis of microRNA target sites was performed using TargetScan Human Release 6.2 (http://www.targetscan.org/). Oligonucleotide pairs were designed to contain wild-type or mutant putative miRNA target sequences in 3′-UTR of PPP2R2A, with proper overhangs and an internal KpnI site for clone confirmation. Annealing and ligating these pairs into the pmirGLO Dual-Luciferase miRNA Target Expression Vector maintained the miRNA target region in the correct 5′ to 3′ orientation. Oligonucleotide pairs were annealed (95°C for 3 min, cooled to 37°C over 60 min and kept at 4°C for 30 min), ligated with the SacI-XbaI digested and gel-purified pmirGLO vector, and transformed into* E. coli* DH5*α*. The positive clones were identified by digesting miniprep-purified DNA with KpnI and verified by sequencing. Cos-7 cells plated on 24-well plates were cotransfected with 50 nmol of either miR-136 mimics or NC oligos and with 200 ng reporter plasmid containing either wild-type or mutant target site using Lipofectamine 2000 Transfection Reagent according to the manufacturer's instructions. Cells were lysed and the relative luciferase activities were quantified at 48 h after transfection using Dual Glo Luciferase Assay System (Promega, WI, USA). All transfections were carried out in triplicate. The oligonucleotide sequences used for each reporter plasmid construction are listed in Table 1.

### 2.7. Western Blot

Protein was harvested using RIPA lysis buffer (Dingguo, Beijing, China) supplemented with 0.1 mmol PMSF, diluted with 5 × RSB, and denatured at 95°C for 10 min. Protein lysates were separated by 10% SDS-PAGE and transferred to PVDF membranes; the membranes were blocked in 5% nonfat milk for 1 h and then incubated with mouse anti-PPP2R2A (1 : 1000, CST, MA, USA) and mouse anti-GAPDH (1 : 5000, KangChen, Shanghai, China) antibodies overnight at 4°C. After incubation with HRP-conjugated secondary antibody (1 : 5000, KangChen, Shanghai, China), protein bands were visualized using Amersham ECL Prime Western Blotting Detection Reagent (GE Healthcare, NJ, USA) on Fujifilm LAS-3000 Imager and quantified by Image J.

### 2.8. Statistical Analysis

Data were expressed as the mean ± SD from at least three independent experiments. Student's* t*-test and one-way ANOVA were used to compare the differences between groups. All statistical analyses were performed using SPSS 16.0 software (SPSS Inc., USA). *P* < 0.05 was considered statistically significant.

## 3. Results

### 3.1. miR-136 Was Downregulated by TGF-*β*1 in HaCaT and NHEK Cells

To investigate miR-136 expression changes during proliferation regulation of TGF-*β*1, we performed quantitative real-time PCR assay to measure miR-136 in keratinocytes treated with different concentration of TGF-*β*1. The result showed that the expression level of miR-136 in HaCaT decreased to 0.19-fold at 48 h after TGF-*β*1 treatment at 2 ng/mL and 0.13-fold for 5 ng/mL TGF-*β*1 (Figure 1(a)). To further confirm this result, we isolated and cultured primary epidermal keratinocytes from normal human skin. The results showed that miR-136 was also significantly downregulated by TGF-*β*1 treatment in NHEK (Figure 1(b)).

### 3.2. miR-136 Suppression by TGF-*β*1 Was Smad3-Dependent

It was reported that Smad2/3 signaling as well as downstream gene targets such as PAI-1 expression is required for TGF-*β* mediated cytostasis in HaCaT cells [19, 20]. To investigate whether canonical Smad2/3 signaling is required for miR-136 repression during TGF-*β*1-induced proliferation arrest in keratinocytes, HaCaT cells were transfected with Smad3 siRNA for 24 h and then treated with 2 ng/mL TGF-*β*1 for 48 h. By quantitative real-time PCR, the mRNA level of Smad3 was decreased to 0.2-fold at 48 h after transfection (Figure 1(c)), and in Smad3-silenced HaCaT cells, TGF-*β*1 treatment showed little effect on miR-136 expression (Figure 1(d)). These results indicated that miR-136 was suppressed by TGF-*β*1 in a Smad3-dependent manner in HaCaT cells.

### 3.3. Overexpression of miR-136 Overcomes TGF-*β*1-Induced Proliferation Arrest

Previous studies showed that TGF-*β*1 inhibited cell proliferation in keratinocytes [21]; to investigate whether forced expression of miR-136 is able to modulate TGF-*β*1-induced proliferation arrest of keratinocytes, HaCaT cells were transfected with miR-136 mimics or miR-NC and subsequently stimulated with 2 ng/mL TGF-*β*1 for 72 h. Successful increased expression of miR-136 was confirmed by qRT-PCR (Figure 2(a)). The results of cell proliferation assay showed that TGF-*β*1 treatment inhibited HaCaT cells proliferation effectively and led to >20% proliferation suppression (Figure 2(b)). Moreover, transfection of miR-136 mimics could negatively regulate the proliferation inhibition of TGF-*β*1 and caused 29% proliferation enhancement. As shown in Figure 2(c), the cell subpopulation in S phase was obviously decreased in TGF-*β*1 treated cells compared with the control group, while the cell number in S phase was significantly increased in cells transfected with miR-136 mimics versus miR-NC group. Taken together, these findings indicated that miR-136 might act as a modulator of TGF-*β*1-induced proliferation arrest in keratinocytes.

### 3.4. PPP2R2A Was a Direct Target of miR-136

To elucidate the underlying mechanisms by which miR-136 exerts its function, we explored miR-136 targets using the TargetScan bioinformatics algorithm. Our analysis revealed that PPP2R2A was a potential target of miR-136 based on putative conserved target sequences at positions 149–155, 712–719, and 1471–1478 of the PPP2R2A 3′-UTR (Figure 3(a)). To further examine whether miR-136 directly targets PPP2R2A, the luciferase reporters containing wild-type or mutant predicted miR-136 binding sites were cotransfected with miR-136 mimics or NC into Cos-7 cells. Luciferase assays were applied 48 h after transfection and the results showed that, compared to NC, transfection with miR-136 resulted in a significant decrease in renilla/firefly luciferase activity of wild-type site 1 and site 2 reporter (Figures 3(b) and 3(c)), while there was no significant decrease of wild-type site 3 reporter (Figure 3(d)). These results suggested that miR-136 repressed PPP2R2A through 2 specific 3′-UTR binding sites at positions 149–155 and 712–719. Notably, the expression of PPP2R2A in HaCaT cells substantially decreased at 48 h after miR-136 transfection (Figure 3(e)). Taken together, these results indicated that miR-136 negatively regulated PPP2R2A in a posttranscriptional manner in HaCaT cells.

### 3.5. PPP2R2A Was Involved in TGF-*β*1-Induced Proliferation Arrest

To further establish whether the counteraction of miR-136 overexpression against TGF-*β*1-induced proliferation arrest is mediated by repression of PPP2R2A, the expression of PPP2R2A in HaCaT cells treated with 2 ng/mL TGF-*β*1 for 48 h was analyzed by Western blot and the proliferation of PPP2R2A knockdown HaCaT cells stimulated with TGF-*β*1 was assessed by proliferation assay and flow cytometry. As shown in Figures 4(a) and 4(b), PPP2R2A in HaCaT cells was upregulated to about 2-fold by 2 ng/mL TGF-*β*1 treatment for 48 hours, and in Figures 4(c) and 4(d), knockdown of PPP2R2A clearly counteracted the proliferation arrest induced by TGF-*β*1. In addition, the reduction of cell cycle progression at G1/S transition induced by TGF-*β*1 was abrogated in PPP2R2A knockdown HaCaT cells. The effects of PPP2R2A knockdown were similar to those induced by miR-136 overexpression. Taken together, these findings indicated that PPP2R2A was a functionally important target of miR-136 and was involved in the TGF-*β*1 regulated proliferation of HaCaT cells.

## 4. Discussion

Wound healing is a complex biological process, during which keratinocyte proliferation and migration are crucial steps for the rapid closure of the epidermis. TGF-*β*1 causes wound margin contraction at the early stage of wound healing and it is responsible for scar formation [22]. These processes are controlled by a network of biomolecules in a spatiotemporal manner. Several recent reports have indicated that miRNAs are involved in regulating keratinocyte proliferation during wound healing [10–14]. Here, we aimed to clarify the biological role of miR-136 in keratinocytes proliferation regulation by TGF-*β*1. The experiments showed significant reduction of miR-136 in keratinocytes treated with TGF-*β*1 and canonical Smad2/3 signaling pathway was involved. Reintroduction of miR-136 by transient transfection, as well as silencing by siRNA of target PPP2R2A, blocked TGF-*β*1-induced proliferation arrest and increased the percentage of keratinocytes in the S phase of the cell cycle, while reducing the percentage of those in the G0/G1 phase. Our results supported the notion that TGF-*β*1-induced proliferation arrest was partially mediated by miR-136 reduction in HaCaT cells.

There are several reports that miR-136 was implicated in cell proliferation and played different roles in different types of cells. miR-136 is proposed to be a tumor suppressor in glioma and is capable of targeting the antiapoptosis genes AEG-1 and BCL-2 [23]. However, miR-136 was found to target tumor suppressor PTEN in breast cancer cells [24]. Recently, results of others indicated that miR-136 enhanced phosphorylation of Erk1/2 through inhibition of PPP2R2A expression to promoted cell proliferation in human non-small cell lung cancer, and the sequence at position 149–155 of the PPP2R2A 3′-UTR was determined to be the target site of miR-136 [25]. In this study, we clarified miR-136 suppressed PPP2R2A expression by directly targeting two conserved regions at positions 149–155 and 712–719 in its 3′-UTR. Furthermore, the protein level of PPP2R2A was significantly reduced by miR-136 mimics transfection in HaCaT cells. Therefore, we proposed that, in the presence of TGF-*β*1, miR-136 was a positive modulator of keratinocytes proliferation and PPP2R2A was a functional target of miR-136 via binding to its 3′-UTR region.

In conclusion, our results indicated that the miR-136 treatment bypassed TGF-*β*1-induced proliferation arrest, at least partially through downregulation of PPP2R2A expression (Figure 5). Our data suggested that modulation of keratinocytes proliferation by miR-136 depends on the cellular environment, especially in the presence of TGF-*β*1, which likely has major effects on the expression of miR-136 target gene PPP2R2A. Further studies are needed to determine whether miR-136 based therapeutic strategies could be exploited to protect keratinocytes proliferation and function in the condition of enhanced TGF-*β*1 during wound healing.

## Figures and Tables

**Figure 1:** miR-136 was downregulated by TGF-*β*1 in a Smad3-dependent manner in HaCaT and NHEK cells. The relative expression levels of miR-136 were determined by quantitative real-time PCR. (a) The expression of miR-136 was downregulated in HaCaT cells treated with 2 ng/mL or 5 ng/mL TGF-*β*1 for 48 h. (b) Downregulation of miR-136 was confirmed in NHEK treated with TGF-*β*1 at the same concentrations and time point. (c) Smad3 silencing by siRNA was verified by quantitative real-time PCR. (d) TGF-*β*1-induced miR-136 repression was counteracted by Smad3 knockdown. Data were presented as mean ± SD values from three independent experiments. Bars indicate SD. ^*^ *P* < 0.05.

**Figure 2:** Overexpression of miR-136 overcame TGF-*β*1-induced proliferation arrest. HaCaT cells were transfected with miR-136 mimics or NC. (a) The miR-136 level in HaCaT cells transfected with miR-136 mimics for 72 h was verified by qRT-PCR. (b) Proliferation assays in HaCaT cells stimulated with 2 ng/mL TGF-*β*1 for 24 h. (c) Flow cytometry analysis revealed the cell cycle distribution. Bars indicate SD. ^*^ *P* < 0.05.

**Figure 3:** PPP2R2A was a direct target of miR-136. (a) There were three potential miR-136 binding sites in PPP2R2A 3′-UTR based on the TargetScan database; the conservation of the miR-136 binding seed regions among different species was shown in shading and mutations were shown in italics. Fragments containing wild-type (wt) or mutant (mut) miR-136 binding sites in human PPP2R2A 3′-UTR were cloned downstream of the luciferase reporter gene separately. ((b)–(d)) Luciferase reporter assay (*n* = 3 for each group). Cos-7 cells were cotransfected with a 3′-UTR reporter construct and the miR-136 mimics or miR-NC, and the results showed that site 1 and site 2 were the direct targets of miR-136. Luciferase activity/renilla activity was applied as the baseline control for the experiments using the same reporter. Data represent mean ± SD. ^*^ *P* < 0.05. (e) Western blot analyses of PPP2R2A expression in HaCaT cells transfected with miR-136 mimics or miR-NC. GAPDH was used as loading control.

**Figure 4:** PPP2R2A was involved in TGF-*β*1-induced proliferation arrest in HaCaT cells. (a) Western blot analysis of PPP2R2A expression in response to TGF-*β*1 treatment. GAPDH was used as internal control. (b) Three independent results of Western blot were quantified by Image J. (c) PPP2R2A silencing was verified by quantitative real-time PCR. (d) Determination of cell viability with Cell Counting Kit-8. (e) Flow cytometry analysis of the cell cycle. Bars indicate SD. ^*^ *P* < 0.05.

**Figure 5:** Schematic representation summarizing the roles of miR-136 and PPP2R2A during TGF-*β*1-induced proliferation arrest. See text for details.

**Table 1:** Oligonucleotides for dual-luciferase reporter assays. All oligonucleotides for 3 target sites were designed with proper overhangs for SacI and XbaI digestion. Mutation sites were shown in italics and KpnI restriction enzyme sites were shown in bold.

Name	Oligonucleotides sequence
wt site 1, sense	5′-C**GGTACC**CAACACATTGTTATAGCTACATGGAGAAAGCTT-3′
wt site 1, antisense	5′-CTAGAAGCTTTCTCCATGTAGCTATAACAATGTGTTG**GGTACC**GAGCT-3′
mut site 1, sense	5′-C**GGTACC**CAACACATTGTTATAGCTAC*GGAACT*AAAGCTT-3′
mut site 1, antisense	5′-CTAGAAGCTTT*AGTTCC*GTAGCTATAACAATGTGTTG**GGTACC**GAGCT-3′
wt site 2, sense	5′-C**GGTACC**ACTGAATAAAAGTGACAAAGAATGGAGAATCTGT-3′
wt site 2, antisense	5′-CTAGACAGATTCTCCATTCTTTGTCACTTTTATTCAGT**GGTACC**GAGCT-3′
mut site 2, sense	5′-C**GGTACC**ACTGAATAAAAGTGACAAAG*CGGAACT*AATCTGT-3′
mut site 2, antisense	5′-CTAGACAGATT*AGTTCCG*CTTTGTCACTTTTATTCAGT**GGTACC**GAGCT-3′
wt site 3, sense	5′-C**GGTACC**GTCAGTCTTGCAGAAACTTTAATGGAGAAGAAAT-3′
wt site 3, antisense	5′-CTAGATTTCTTCTCCATTAAAGTTTCTGCAAGACTGAC**GGTACC**GAGCT-3′
mut site 3, sense	5′-C**GGTACC**GTCAGTCTTGCAGAAACTTT*CGGAACT*AAGAAAT-3′
mut site 3, antisense	5′-CTAGATTTCTT*AGTTCCG*AAAGTTTCTGCAAGACTGAC**GGTACC**GAGCT-3′
